# Indonesian Migrant Workers: The Migration Process and Vulnerability to COVID-19

**DOI:** 10.1155/2022/2563684

**Published:** 2022-06-15

**Authors:** Aswatini Anaf, Fitranita Ibnu, Haning Romdiati, Mita Noveria

**Affiliations:** Research Center for Population-National Research and Innovation Agency, Jakarta, Indonesia

## Abstract

Indonesia is one of the largest sources of migrant workers in Southeast Asia. Presently, these workers are vulnerable to COVID-19 due to the prolonged migration process, which requires them to relocate from their villages to another country and back to Indonesia on completion of their working contract. Therefore, this study describes and discusses the vulnerability of Indonesian migrant workers (IMWs) to the pandemic at various phases of the migration process. It is related to the implementation and practice of health protocols, ignorance and indifference to the dangers and transmission of the virus, and also to the national vaccination program. The analysis is based on the review of literature studies, such as studies related to the topic, international and national regulations on migrant workers, and official data and statistics published by the Indonesian government. The materials and data were collected from search engines such as Google Search and Google Scholar and also relevant published reports available. Several policies have been implemented by the government of Indonesia and other destination countries where the prospective IMWs intend to work, to protect and prevent the transmission of COVID-19. However, there is still a contagion among IMWs willing to leave abroad and those returning home after completing their employment contract. Therefore, both countries need to be responsible for each migration process, specifically related to providing health protection, increasing awareness of the danger and transmission of the virus, and applying polymerase chain reaction (PCR) tests and COVID-19 vaccination for migrant workers.

## 1. Introduction

Migration is a global phenomenon that influences the population's health [1] and geographical limit due to disease transmission, such as in the case of the COVID-19 pandemic [2]. On March 11, 2020, the World Health Organization (WHO) declared this outbreak as a global pandemic due to its rapid spread [3]. One effort adopted by various countries was to restrict the international population's mobility [3, 4], which inevitably affected the movement of migrant workers.

Indonesia plays an important role as a labour-sending nation in Southeast Asia, with a significant number of IMWs, persons who cross international borders for work, found in Asian and Middle Eastern Countries. In 2019, it was reported that approximately 3.7 million Indonesians worked abroad [4]. Globalization with increased interconnectivity and dependency on both the sending and receiving countries boosts international labour migration and enhances economic growth. The governments' policy in several countries worldwide on the restriction of international population mobility due to the COVID-19 pandemic has also influenced IMW placement.

IMWs are a group of people vulnerable to the pandemic due to the lengthy migration process they have to undergo, which puts them at risk of transmission. This study aims to explore and examine the vulnerability of IMWs to COVID-19 from the preparatory phase in their home country to their return, at the end of their working term abroad. Vulnerability to COVID-19 is defined as being exposed to the possibility of contracting the virus in each phase during the migration process. This analysis is based on the review of literature studies and documents, namely, studies related to the topic, international conventions on the protection of migrant workers, official data, statistics, and documents, and regulations published by the Indonesian government on the deployment and protection of Indonesian migrant workers. The materials are obtained from search engines such as Google Search and Google Scholar and relevant published reports available.

### 1.1. Indonesian Migrant Workers and COVID-19

Evidence showed that COVID-19 spreads as a result of direct or close contact with infected people through mouth and nose secretions and indirect causes, such as through contaminated objects or surfaces [5].

- It occurs mainly between people that are in close contact with each other, typically within 1 metre (short-range). A person is infected when aerosols or droplets containing the virus are inhaled or comes in direct contact with the eyes, nose, or mouth.
- In poorly ventilated or crowded indoor areas, because people tend to spend more extended periods in such settings. This is because aerosols remain suspended in the air or travel farther than 1 metre (long-range).
- By touching their eyes, nose, or mouth without washing or sanitizing their hands after coming in contact with contaminated surfaces.

It is important to practice health protocols to reduce an individual's chances of getting infected or spreading the virus [6]. However, adequate protection is achieved through vaccination, which protects the individual from contracting the virus. Vaccination has been shown to contribute to reducing death rates, severe illness, and transmission of COVID-19 [7]. One of the efforts to prevent the spread of the SARS-CoV-2 virus is by limiting human mobility both internally and externally, which includes international labour. Migrant workers are vulnerable to COVID-19 due to the lengthy migration process, which exposes them to factors potentially related to the virus transmission. This situation is associated with the inability to implement health protocols, either caused by self-negligence or due to the unavailability of necessary supporting facilities for their protection and also the vaccination program, specifically in the country of origin.

On April 13, 2020, the Indonesian government declared the COVID-19 outbreak as a nonnatural, national disaster [8]. According to a 2021 survey, the total number of COVID-19-infected cases in Indonesia on December 26, 2021, was approximately 4.26 million. Furthermore, the number of active cases decreased from 574,135 in July 24, 2021 (the highest in 2021) to 4,655 in December 2021 [9]. The Indonesian government, in an effort to prevent the spread and transmission of the virus, developed and promoted a health protocol that contains certain guidelines and recommendations, known as 3M, which constitutes wearing a mask, washing hands with soap under running water, and maintaining social distancing [10]. This policy was further expanded to 5M with 2 additional recommendations, namely, avoiding crowds and reducing mobility [11]. The Indonesian government also implemented a COVID-19 vaccination program for the entire population, which started on January 13, 2021 [12]. Presently, there is no specific policy for COVID-19 vaccination for prospective migrant workers, the vaccination program also applied to them.

Indonesia is the second country with the highest number of people migrating to other nations in Southeast Asia after the Philippines [13–15]. In 2016, approximately 9 million Indonesians worked as documented and undocumented workers [16]. The important destination countries for IMWs are Malaysia, Taiwan, Saudi Arabia, Hong Kong, and Singapore, as shown in Table 1, and they are also exposed to COVID-19 in varying severities. Therefore, IMWs are also at risk to infectious diseases during their time working abroad.

The Indonesian government stated that IMWs will be repatriated in line with health protocols, which also applied to all those who entered the country during the pandemic [20]. This procedure will filter the IMWs infected with the virus, either while in the countries where they worked or during their travel back to Indonesia. Some data showed that among the returning IMWs, many workers were infected with COVID-19, based on the polymerase chain reaction (PCR) test on their arrival. For example, among 14 thousand IMWs repatriated from Malaysia, between January and April 2021, 200 were infected by COVID-19, based on PCR tests in Batam port (Riau Islands Province) on their arrival in Indonesia [21]. On September 29, 2021, approximately 1,892 IMWs from a total of 27,882 workers who arrived in Batam from Malaysia and Singapore were found infected [22]. As of September 11, 2021, the East Java Provincial Health Office has conducted PCR tests on 34,840 returning migrant workers and 2,188 people tested positive for COVID-19 [23]. All the returned IMWs are likely to be infected while working abroad or during their return travel to Indonesia.

In terms of place of origin, three main provinces in Java Island, namely, West Java, Central Java, and East Java were the largest senders of IMWs, as shown in Table 1 and Aswatini et al. [24]. These three provinces are also known as those with the highest number of COVID-19 cases in Indonesia [25]. Therefore, IMWs that return home are also at risk, due to the high number of cases in their home and working areas.

Data collected from 2016 to 2021 showed that the majority of IMWs education level is low, specifically elementary school and junior high school graduates. This implies that their major types of work include domestic helpers and caregivers, which are informal sector jobs, as shown in Table 1. Low educational level is one of the causes of inadequate knowledge about COVID-19; therefore, it is believed that IMWs do not have sufficient insight to keep themselves from getting infected. The type of work performed by IMWs, such as caregivers, is prone to infection because they may have to accompany their employer to the hospital and be with them also causing direct contact with people outside the workplace. Furthermore, the migration phases, which require them to go through from their place of origin to destination countries and return, indicated that they are exposed to the possibility of contracting the virus.

## 2. Materials and Methods

International Labour Organization Migration for Employment Convention (revised) 1949 (no. 97, article 5) [26] stated that for migrant workers and their families to be in a reasonable health condition, they need to enjoy adequate medical attention and good hygienic conditions at the time of departure, during the journey, and upon arrival to the destination countries. These three phases of the migration process demonstrate the importance of migrant workers and accompanying family members to be in good health in the destination country without considering their health conditions.

The United Nations International Convention on the Protection of the Rights of All Migrant Workers and Members of Their Families [27] convinced that appropriate international protection is needed for their fundamental human rights, including health protection, as stated in Part III, Article 28, of the convention. It describes all the rights applied during the entire migration process of migrant workers and members of their families, which comprises preparation for departure, transit, and the entire period of stay and remunerated activity in the state of employment as well as return to their habitual residence (Part I, Article 1 of the convention). The protection guaranteed in United Nations Convention is broader than the ILO because it includes the preparation process in the country of origin until the migrant workers returns. It is clear that the majority will only live and work in the destination country for a certain period of time, and after completing their employment contracts, they return home.

According to Law Number 18 of 2017 concerning the protection of Indonesian migrant workers and their families [28], the protection should cover pre- and post-work phases. The purpose of the law to ensure the fulfilment of human rights as an Indonesian citizen and IMWs and cover the legal, economic, and social protection. The social protection also covered the health insurance in the three phases as indicated in Article 15, paragraph 2. The prework phase is defined as the entire activity from registration to departure. The work phase is the whole activity of the IMW's and their family members, while the after-work phase is the whole activity after they return to their home regions.

In the context of contemporary migration, Zimmerman et al. [29] stated that migration is a complex process that may occur within or across national borders. With respect to the health risks faced by migrants, they described that it consists of predeparture, travel, destination, interception, and return phases. The predeparture and travel phases cover the time before individuals left their place of origin and the timeframe between their place of origin and destination. The destination phase is when individuals settle in their destination countries, while interception applies to the situation of temporary detention, and the return phase is when individuals return to their country of origin.

From the above review, it is obvious that the migration process started from the migrants' place of origin to their return after completing their working period abroad. The migration phase is an important factor to be considered in providing migrants with health protection including infectious disease transmission [29–31]. Based on the aforementioned review, it can be concluded that for the purpose of analysing the IMWs' vulnerability to COVID-19, the migration process consists of four phases as follows:

1. *Preparatory Phase*. This phase comprises the recruitment and predeparture period, in the country of origin.
2. *Travel and Transit Phases*. This period starts from migrant workers' departure from their home country to destination countries over a short period.
3. *Destination Phase*. It starts from migrant workers' arrival and the entire period of stay and work in destination countries.
4. *Return Phase*. The period starts when the migrant workers leave their host countries and return to their state of origin.

The analysis adopted a two-stage review. The first developed framework of the migration process for IMWs consists of four phases. The second determined the vulnerability of IMWs to the virus in each migration phase by exploring and investigating the available literature and data on the situation of IMWs. These include published study results, government documents, websites of relevant ministries and agencies, statistical data on IMWs, and COVID-19 protocols released by the Indonesian government and related studies.

## 3. Indonesian Migrant Workers' Vulnerability to COVID-19

### 3.1. Preparatory Phase

The preparatory phase comprises the recruitment and predeparture process, that is, the period before prospective migrant workers depart from their country of origin. According to Indonesian government Regulation Number 10, concerning Procedures for Placement of Indonesian Migrant Workers, article 9, this phase includes 10 activities, namely, (1) dissemination of information, (2) registration, (3) selection, (4) health and psychological examinations, (5) signing a placement agreement, (6) social security membership registration, (7) processing a work visa, (8) implementation of predeparture orientation, (9) signing the work agreement, and (10) departure [32]. Some of these activities expose prospective IMWs to COVID-19, such as the dissemination of information concerning employment conditions abroad, obtaining registration documents, and predeparture activities.

The potential spread of the virus increases significantly during the dissemination of information regarding employment conditions abroad due to the gathering of prospective IMWs in a particular place. Overcrowding becomes an inevitable condition because of the difficulty in maintaining social distancing. This condition is exacerbated by the lack of awareness (dangers and transmission) concerning the prevention of COVID-19. The majority of the prospective IMWs are poorly educated (Table 1); therefore, it seems like they tend to be ignorant of the health protocols. Several studies reported that properly educated individuals usually practice the health protocols to guard against the spread of the virus [33–35]. In addition, a lack of knowledge and understanding is also related to noncompliance with wearing masks [36]. These results could be because of participants with higher educational levels having better comprehension of COVID-19 transmission compared with their counterparts. A study on “Knowledge and Awareness of COVID-19 among IMWs in the Greater China Region” found that those with elementary or junior high school education were less likely to correctly answer questions on virus transmission route, drug and vaccine availability, and quarantine periods compared with their peers with higher educational backgrounds [37]. Aside from the difficulty in avoiding crowds, the dissemination of information also causes prospective IMWs' inability to reduce mobility, which is one of the efforts to curb the spread of the virus.

The vulnerability to COVID-19 transmission also occurs during the process of obtaining the required documents for registration. This is because prospective IMWs have to visit several offices, for example, the Village Office and Office of Population and Civil Registration, to apply for an electronic identity card (e-KTP). The possibility of contracting the virus in this stage is quite high, as large crowds are unavoidable, making it difficult to maintain physical distance. The vulnerability of prospective IMWs to this disease increases supposing the public service offices provide limited or no hand washing facilities, including soap and running water.

IMWs from sending areas with high cases of COVID-19, such as East, Central, and West Java provinces (up to March 2020, the number of IMWs placed from the provinces of East, Central, and West Java was 13.2, 11.8, and 11.7 thousand, respectively [38–40], while the cases of the population infected with COVID-19 in those three provinces at the same time were 93 (East Java), 93 (Central Java), and 198 persons (West Java) [41]. These provinces were the second (West Java) and the fourth (East and Central Java) of the COVID-19 epicentre, apart from DKI Jakarta (747 persons) and the Banten province (142 persons), are likely to be more vulnerable to virus transmission compared to those in other regions. The more the recorded cases, the more susceptible prospective IMWs are to the virus transmission. As mentioned earlier, the poor education and understanding of prospective migrant workers regarding the dangers of the virus and its transmission contribute to their ignorance of the use of health protocols, thereby leading to high vulnerability. The educational factors and government policies not enacted at the village level cause ignorance or low knowledge on the dangers and ways of preventing transmission, for example, Indonesia has established Government Regulation No.1 of 2020 as a reference for agencies, both at the provincial to district levels, in dealing with the pandemic by implementing health protocols to curb the spread of the virus [42]. However, rural communities poorly understand these policies, especially those in remote villages, due to the lack of socialization and awareness on COVID-19 [43].

The registration process is performed online, which is a relatively safe initiative. At some point, it became a concern to the ILO, which stated that recruitment practices need to adapt to the COVID-19 preventive measures quickly. Some of these include shifting to online modalities and adopting safe and fair recruitment practices once travel restrictions are lifted [44]. This is because the health, well-being, and safety of job seekers and migrant workers is a priority for labour recruiters during this crisis [45]. However, IMWs in villages with limited Internet networks, poor communication services, inadequate educational backgrounds, and mediocre economic conditions tend to find online registration difficult [46–48]. Hence, due to economic constraints [49, 50], it is believed that they are unable to access private internet networks; therefore, they have no choice but to use public telecommunication services. Unfortunately, the use of these facilities involves a queue, which triggers the spread of the virus. These are some of the obstacles faced by prospective IMWs in implementing health protocols, especially in maintaining social distancing.

To work abroad, they are required to adhere to a series of preparatory activities before departure (Indonesian Government Regulation No. 10 of 2017) [51]. In conjunction with the Indonesian Migrant Worker Placement Company, the government at the district or city level also engages in these schemes. Before the pandemic, participating in training activities and preparing for departure require the prospective IMWs to stay in a shelter. Generally, the residents exceeded the stated capacity, which resulted in unhealthy living conditions characterized by poor ventilation, limited facilities for clean water, and environmental sanitation [52]. Under these circumstances, infectious diseases are difficult to control; therefore, they tend to spread quickly. During this pandemic, these shelter conditions are a source of transmission because they are not conducive for social distancing and a healthy lifestyle. Therefore, to curb the spread of the virus, these facilities need to be adjusted to adhere to physical and social distancing requirements that are extremely necessary [53].

Prior to departure, the prospective IMWs have to attend educational and training activities to obtain work competency certificates according to the type of job sought abroad (Government Regulation No. 18 of 2017) [51]. During the pandemic, the government announced that awareness and training sessions have to be carried out using a blended learning mechanism that involves a combination of online and offline or face-to-face interactions [54]. This reflects that prospective IMWs tend to be vulnerable to COVID-19 transmission. Therefore, the training method requires adherence to social distancing and wearing masks.

In preparation for departure, the health and psychological diagnosis of the prospective IMWs is carried out in government-approved facilities (Government Regulation No. 10 of 2020) [51]. These are in the form of complete physical and mental examinations performed by doctors (Minister of Manpower, Decree No.294 of 2020) [55]. This investigation aims to ensure that they do not infect the population in the host country. Furthermore, due to the pandemic, medical examinations require a polymerase chain reaction (PCR) test commonly used to diagnose COVID-19 in government-approved health facilities. The cost of the PCR test is free of charge for prospective IMWs [56]. During this activity, the risk of contracting the virus is quite slim, since the organizers are government agencies that generally adhere to the proper implementation of health protocols. Furthermore, during the predeparture orientation period, there is a need to sign a work contract with the IMWPA. In the final stage, the migrants are less susceptible to COVID-19 simply because the organizers enforced strict health protocols. In the preparatory phase, the most recent activity is the IMWs' departure from the shelter to the airport by bus. During this trip, they are invulnerable to virus transmission because all have undergone PCR examinations.

In addition to having a negative PCR test result, the prospective IMWs must ensure they receive complete vaccination comprising of two doses and are validated by the Indonesian Ministry of Health. Although there is no specific policy regarding vaccination for them, it is an effort to minimize the level of COVID-19 transmission and raise the immune system to reduce the number of cases [57].

The Indonesian Ministry of Manpower partners with the Indonesian Ministry of Health to ensure appropriate support for COVID-19 vaccination access for the prospective IMWs. The vaccines are provided by the government, free of charge [58], and the prospective IMWs can get a certificate issued by the Ministry of Health after receiving a complete dose to fulfil several administrative requirements [59]. These include (1) a cover letter from IMWPA/IMWP/Ministry of Manpower which contains a list of the prospective IMWs' names, ID cards, passport numbers, and addresses, (2) a copy of their identities stored in computers, (3) a copy of their identity page, (4) a copy of their ID card, and (5) a print-out of the vaccination certificate in the format of application of COVID-19 protection care (*Peduli Lindungi*).

Several destination countries such as Taiwan [60] and Hong Kong [61] by August 30, 2021, have mandated the presentation of a COVID-19 vaccine certificate as one of the requirements for workers seeking entry. Fully vaccinated foreign domestic helpers (FDHs) who were fully vaccinated in Indonesia are allowed to work in Hong Kong [61]. The Sinovac-CoronaVac COVID-19 vaccine, which is commonly used in Indonesia is not accepted by certain destination countries of the IMWs, such as Taiwan [62]. In response to this denial, the Ministry of Manpower of Indonesia has made efforts to provide other types of vaccines to prospective migrant workers, such as AstraZeneca [63].

Only a small number of IMWs received the vaccine before being dispatched by the IMWPA. Data show that as of August 30, 2021, as many as 11,375 prospective IMWs received their complete vaccinations [62], and by December 2021, approximately 61,186 needed vaccination due to their plan to work abroad [59]. This vaccine is very important not only to protect the IMWs from the virus transmission, but also in order to eradicate stigmatization on the IMWs who are often considered carriers.

### 3.2. Travel and Transit Phases

The travel and transit phases involve a journey from the migrants' state of origin to their destination countries, specifically the workplaces. They use various transportation modes to get to the countries. Besides the major means, such as ships and airplanes, IMWs are also conveyed in buses and trains to the seaport or airport. Many migrant workers undertake direct trips to their destinations, while others are placed in transit at any particular time, depending on the schedule of their connecting flights or voyages. These phases are the shortest periods in the migration process undergone by the IMWs, after carefully planning to avoid the risk of infectious disease and exposure during the journey to their destinations [30]. One of the ways to minimize risk of possible infection is by ensuring IMWs head straight to their designated workplaces once they reach their destination countries to avoid crowded areas, which in turn prevents them from contracting infectious diseases.

Several destination countries, such as Hong Kong, request migrant workers, including IMWs, to present several documents while boarding a flight. These include (a) a recognised vaccination record issued by the Indonesian authorities, (b) a valid employment visa for FDHs issued by the Immigration Department (ImmD) of Hong Kong, (c) negative result proof of a polymerase chain reaction-based nucleic acid test for COVID-19 with specimen collected within 72 hours before the scheduled time of departure, and (d) confirmation of room reservation at a DQF for not less than 21 nights starting from the day of arrival in Hong Kong [61].

Irrespective of the fact that IMWs are reported to have a negative status before departure, they are susceptible to contagious diseases during the trip. The COVID-19 pandemic is caused by SARS-CoV-2 which is the third adaptation of a contagious virus following the severe acute respiratory syndrome coronavirus (SARS-CoV) and the Middle East respiratory syndrome virus (MERS-CoV) [64]. Those that congregate in close proximity and join other passengers on any public transport mode are vulnerable to COVID-19. Pathogens tend to be transferred from those across different zones [29]. It is impossible to maintain physical distancing among passengers, making them vulnerable to any transmissible diseases, including COVID-19. In addition, when they arrive at the ports, migrant workers join the crowd while waiting to board the primary vehicle, which makes them prone to contracting other contagious diseases. Migrant workers, especially those travelling by airplane, inhale recirculated air during the journey [65]. Although there is few evidence to this effect, there is a long-held belief in some circles that respiratory infections are commonly transmitted onboard aircrafts [66]. Therefore, in the context of contagious diseases such as COVID-19, IMWs are assumed to be prone to the virus while on the airplane.

In case where they have to transit at any of the ports, which means having to alight the aircraft or ship and wait, before embarking on the journey, they are amidst a crowd with passengers from other regions. There is a possibility of suspected disease carriers among the crowd, and IMWs tend to be infected. During such situations, it is essential for them to strictly adhere to the health protocols related to preventing the virus, such as always using their face masks, washing hands as often as possible to keep them clean, and maintaining social distancing from others. Apart from adequate knowledge, self-discipline is strongly needed to prevent the spread of COVID-19. It is paramount that they have spare face masks and hand sanitizers that are used when needed.

All attempts to prevent IMWs from contracting the virus have to be supported by the ports where they depart and transit by providing all necessary facilities. For example, handwashing equipment needs to be adequately provided in terms of number, availability of clean water and soap or sanitizers, and installed close to the passengers' waiting rooms at all international ports. This urges the passenger to wash their hands regularly, particularly after touching surfaces that are probably contaminated with viruses. Moreover, these ports need to provide waiting rooms to accommodate the passengers in such a manner that they observe social distancing to hinder transmission.

### 3.3. Destination Phase

Each stage of the migration process has specific characteristics related to the transmission of contagious diseases, including COVID-19. In respect to various stages, the longest period is the destination phase. The shortest period of a single contract signed by IMWs is 2 years, with a possibility of extension. Therefore, it is reasonable to speculate that migrant workers are vulnerable to disease transmission throughout the destination phase compared to the other stages. This is especially true for those in high-risk areas, countries, and cities with an increasing number of COVID-19 cases.

This phase involves the arrival of migrant workers at their destinations, where they are taken to their respective workplaces. In the IMWs context, their movement is under national or special parties' arrangement, and the processes are managed by agents that collaborate with the government or private labour-sending agencies. IMWs employed in the formal sector, such as factory workers and institutional caregivers, are taken to dormitories provided by their employers [67]. Moreover, those recruited in the domestic sector, such as housemaids and caregivers, are taken to their places of employment. Occasionally, they are stopped at agents' places before being taken to their final destination. At the agent's place, where they spend only one night, the newly arrived IMWs probably meet other migrant workers from other countries, although this exposes them to the virus.

Many countries have implemented standard procedures in examining the health conditions of travellers, including migrant workers, at sea terminals and airports. A rapid clinical evaluation is performed to screen newly arrived passengers. This helps to prevent the transmission of infectious diseases to the host population [68]. For example, Taiwan has issued 3 regulations for incoming passengers since the pandemic, aside from restricting foreigners from entering the country. Only certain categories of people have been eligible to enter Taiwan since the outbreak. This includes migrant workers that meet all the requirements stipulated by the Taiwan government. The first issued regulation mandates that from June 29, 2020, all foreign nationals need to present a negative COVID-19 test certificate written in English, taken within 3 working days of boarding the flight to Taiwan. Such people also have to be quarantined for 14 days once they enter the country [69].

Following this policy, the second rule was specifically launched for migrant workers, and it took effect from December 10, 2020. The policy reported that after undergoing a 14-day group or home quarantine, they need to be further observed under 7-day self-health management [69]. The employers are expected to provide a place for the migrant workers to be observed for 7 days. During the self-health management period, each of them is expected to stay in an independent room. In circumstances where this is impossible, they need to maintain a distance of 1.5 meters, wear a mask, and ensure the environment is properly sanitized and disinfected.

The recent regulation launched by Taiwan in early 2021 strictly restricted entry into the country. This policy which was implemented on January 15, 2021, mandated that on arrival, the migrants also need to provide proof of the location for their intended quarantine besides the original requirement of providing a COVID-19 reverse transcription-polymerase chain reaction (RT-PCR) test report issued within 3 days of boarding [70]. They need to be kept in a group quarantine facility or hotel. In circumstances where they choose to be quarantined at home, there is a need to ensure that such activity is carried out 1 person per residence.

Taiwan's government regulation on 14-day quarantine in addition to 7-day self-health management benefitted both the host population and migrant workers. These 2 policies aim to curb the transmission of the virus. After completing the quarantine and self-health management period, they are assured of not being infected, thereby, unable to spread the disease to others, mainly those close to them. On the aspect of the migrant workers, their health condition was likely monitored during these processes. However, in circumstances where they are infected with COVID-19, they probably need to obtain medical treatment.

The Indonesian government has also carried out attempts to curb the transmission of this virus. They launched a medical screening health protocol on May 1, 2020, for foreigners on arrival at the seaports and airports in many cities [71]. These include migrant workers that were laid off and forced to travel home due to the lockdown policies in the host countries. According to the health protocol, anyone detected to be infected with SARS-CoV-2 has to be treated for COVID-19. Moreover, those that are not infected are suggested to self-isolate for at least 14 days.

Migrant workers generate public health problems in host countries [4], especially those that are highly dependent on them [72]. At the micro level, this tends to affect other individuals. Migrant workers are threatened by contagious diseases, although on the contrary, assuming they were suffering from such ailments, they tend to transmit it to persons living close to them.

IMWs are mostly employed in the informal and domestic sectors of the host countries. For instance, in Hong Kong and Taiwan, most of them work as domestic staff and caregivers [17–19]. Some IMWs, particularly males and other migrant workers from Southeast Asian countries, such as the Philippines and Vietnam, are usually employed in the fish industry in Taiwan [73]. Furthermore, in Malaysia, some of them work in manufacturing and plantation establishments, besides, a huge number are employed in the domestic sector as housemaids and babysitters. Due to the diverse jobs, IMWs reside in different areas during their stay overseas. Domestic staff and caregivers stay at their employers' houses [74], while those that work in manufacturing industries live in dormitories, either within or outside the factory. Furthermore, plantation workers reside in barracks provided by the company in the vicinity [67]. IMWs that are fish workers in Taiwan spend quality time in the vessels with others.

IMWs are exposed to contagious diseases, such as COVID-19, in various ways throughout the destination phase in host countries. This relates to their living or working conditions, because according to [3] they usually live in crowded environments with limited access to basic needs such as water and hygiene products. For example, the barracks inhabited by IMWs in Malaysia are overcrowded with poorly ventilated and limited sanitation facilities [67]. This inevitably facilitates the transmission of infectious diseases, including COVID-19. Many farmworkers from Mexico and Commonwealth Caribbean countries in Canada live in narrow quarters that are poorly ventilated [75]. In Germany, Romanian farm migrant workers also encounter similar experiences. They live in crowded communal camps in which physical distancing and appropriate sanitation practices are difficult to apply [76].

IMWs living with their employers are also exposed to the pandemic because an infected family member is likely to transmit the disease to others, including housemaids or caregivers. This condition is particularly worsened assuming they are not provided with health insurance and in circumstances where the employers refuse to pay for their medical treatment, IMWs need to bear the costs. Meanwhile, those with insufficient money for medical services, probably because their salaries were remitted to their families, are the most disadvantaged group throughout the pandemic.

Poor living conditions are also experienced by those that work in Gulf. In Kuwait, the few IMWs employed, for instance, live in extremely bad housing conditions, such as cramped and poorly ventilated dormitories with dilapidated toilets shared by everyone and close proximity among the occupants [77]. Such situations are unfavourable in the prevention of COVID-19, as it requires healthy living conditions with adequate clean water for washing hands and showering, as well as a representative space for maintaining appropriate social distancing. In circumstances where a worker becomes infected, it is difficult to isolate the victim because the available space accommodates many people.

A similar situation occurred in Singapore, where relatively three-quarter of new COVID-19 cases were related to low-skilled migrant workers living in dormitories [4]. A study carried out in Singapore from January 30, 2020, to April 30, 2020, reported that 76.7 percent of the confirmed cases were migrant workers living in dormitories [78]. A survey carried out from April 22, 2020, to 26, 2020, revealed that migrant workers living in dilapidated dormitory dwellings constitute 94.6 percent [79]. However, most IMWs in this country work and live with their employers, while a small percentage of those that live in dormitories remain vulnerable to the pandemic.

Vulnerability to COVID-19 also comes from poor working conditions. As mentioned earlier, many IMWs fish workers in Taiwan spend most of their time in the vessels. This makes them vulnerable to the virus, including when they became stranded at the port due to the lockdown policy [73]. They were prohibited from getting off the vessel and asked to stay with the crew. This unfavourable condition made them vulnerable to the virus, combined with the difficulties encountered in terms of access to health services.

Vulnerability to COVID-19 is not only experienced by IMWs that were not laid off. The majority of those that lost their jobs due to the termination of certain economic activities are also susceptible to disease transmission. A survey carried out in 9 IMWs host countries by the Human Right Working Group (HRWG) in collaboration with *Serikat Buruh Migran*, Indonesia (SBMI–Indonesian Labour Migrant Union) and *Jaringan Buruh Migran* (JBM-Migrant Workers Network) in late April 2020, reported that the reduction in income and laid-off workers are among the impacts of the pandemic on such groups [80]. This forced the IMWs to leave their usual residence, such as factory dormitories, searching for alternative dwellings. A reasonable option was to put up with other migrant workers, which lessens the expenditure on accommodation. Typically, they live in crowded places, making them vulnerable to the disease.

Documented IMWs are beneficiaries of health services during their work contract, as long as they pay for the insurance fees. In Taiwan, migrant workers have to pay these fees by themselves. Meanwhile, in Malaysia, employers insured domestic staff through the Foreign Worker Compensation Scheme, which enables them to obtain medical treatment when they suffer from injuries related to work accidents, as stated in the contract letter. Although some receive medical treatment through health insurance coverage, the majority do not have such access [4]. Moreover, medical services related to COVID-19 treatment are not covered by health insurance. In the case of Malaysia, for example, this process only covers medical services caused by related employment injuries.

The Indonesian government has implemented some policies to ensure more protection to IMWs during the destination phase, such as communicating with employers to create flexible working hours without reducing their salary. This decreases the IMWs' time to gather with other employees at work. Those who lost their jobs were provided the necessary funds to return home [81] while they remain practicing health protocols and ensuring negative COVID-19 results based on the PCR test to prevent the spread of COVID-19. Moreover, the Ministry of Foreign Affairs has developed a website portal that enables Indonesian citizens abroad to report their health conditions [82]. Development of the portal is not exclusively a response to the COVID-19 pandemic; however, it will be able to identify Indonesian citizens suffering from the virus.

### 3.4. Return Phase

The return phase is when the migrant workers leave their host countries and return to their state of origin. There are 2 reasons that induce them to leave for their homes. First, they have completed their working contract and do not intend or are not eligible to extend its duration. Secondly, they are forced to return home due to ill health and chronic or terminal diseases [83].

There is a gap in health examinations related to the return phase [83]. Unlike at departure, the screening procedure is not crucial for migrant workers during their home journey. Therefore, it was concluded that it is not necessary for migrant workers. On the contrary, unless the Indonesian Government carries out a medical examination, IMWs tend to import pathogens transmitted to those at home. Besides, those infected in the host country are entitled to medical treatment, as stated in the International Convention on the Protection of the Rights of All Migrant Workers and Members of Their Families (Article 43.1.e). However, since the pandemic is an emerging infectious disease, it is doubtful whether COVID-19 is included in medical treatment coverage.

Returning IMWs infected by the virus constitute health problems for those at home. The individuals close to them are likely to get infected. The Indonesian Government has carried out several attempts to prevent the possible transfer of this virus. According to the implemented health protocols, returning IMWs and other migrants have to undergo the COVID-19 screening procedure on arrival [71]. In cases where symptoms, such as cough and high fever, are detected, they are treated in a government-approved health facility. In addition, both returning IMWs and citizens arriving from overseas are isolated for a certain period.

Many returning IMWs were infected with the virus, which was confirmed on arrival. Data show that from January to April 2020, 200 out of 14.000 IMWs that arrived in Batam, Riau Island province, from Malaysia, for instance, were confirmed cases of COVID-19 [21]. However, it is difficult to determine when they contracted the disease, in Malaysia or during the return trip to their home towns. According to Indonesian regulations, the infected returning IMWs need to be quarantined to curb the spread of the virus. Therefore, they are transferred to the COVID-19 referral hospital in Galang Island, located in Riau Islands province.

## 4. Conclusion

On April 13, 2020, the Indonesian government declared the COVID-19 outbreak a nonnatural national disaster. Generally, to prevent the spread and transmission of this deadly virus, health protocols that contain guidelines and recommendations were developed and promoted. This is known as 5M and based on suggestions for people to practice a healthy lifestyle daily.

The health protocol was implemented during the sending process by the institutions involved in recruitment and placement as well as the IMWs themselves, a group of migrants vulnerable to the virus. Several supporting policies related to implementing the 5M health protocol have been carried out by the government and IMWs recruitment and placement agencies. However, there are still positive cases of the virus among departing and returning due to difficulties in the application of health protocols, lack of supporting facilities or indifference among prospective Indonesian migrant workers, and poor socialization and advocacy on the dangers and ways of COVID-19 transmission.

On January 13, 2021, the government mandated the administration of a COVID-19 vaccination program for the entire population, as well as prospective migrant workers. The PCR test is also an obligation for each prospective IMWs to ensure they leave the country in good health and to those who have just arrived. Preparation is the most important phase in the IMW migration process because it reduces their vulnerability to COVID-19 transmission. Besides the test to detect the infected and the efforts to increase the IMWs' immunity to COVID-19 by vaccination, the preparation phase is a starting point for empowering them to understand the danger and ways of the virus transmission. All these efforts are very useful for their protection when travelling and transiting to their various destinations.

Efforts to reduce the vulnerability of IMWs to the virus are also the concern and responsibility of the Indonesian government and the host countries. PCR tests need to be conducted at the time of departure, arrival to their destinations, and when return. The destination country needs to provide facilities that allow IMWs to implement health protocols, including providing viable lodging for those who do not stay in their employer's home.

The government and private agencies involved in the recruitment and placement process in both Indonesia and other host countries need to advocate for IMWs to be aware of the dangers and transmissions of the virus. The health insurance coverage of IMWs needs to be expanded to cover and guarantee the treatment of the pandemic during every stage of the migration process.

## Figures and Tables

**Table 1:** Some indicators of Indonesian migrant workers (IMWs) deployed to work abroad, 2016–2021.

Indonesian migrant workers' indicators	Year					
	2016	2017	2018	2019	2020	2021
Total number of workers deployed abroad	234,451	262,899	283,640	276,553	113,173	59,053

Sex Percentage of females	62	70	70	69	80	90

Education Percentage with junior high school education and below	68	71	70	64	64	61

Employment sector Percentage of workers working in nonformal jobs	47	55	53	52	67	78

Occupation 3 main occupations (in order)	(1) Caregiver (2) Domestic workers (3) Plantation workers	(1) Domestic workers (2) Caregiver (3) Operator	(1) Domestic workers (2) Caregiver (3) Operator	(1) Domestic workers (2) Caregiver (3) Operator	(1) Domestic workers (2) Caregiver (3) General workers	(1) Domestic workers (2) Caregivers (3) General worker

Province of origin 3 most important provinces of origin (in order)	(1) West Java (2) Central Java (3) East Java	(1) West Java (2) Central Java (3) East Java	(1 West Java (2) Central Java (3) East Java	(1) East Java (2) Central Java (3) West Java	(1) East Java (2) Central Java (3) West Java	(1) East Java (2) Central Java (3) West Java

Destination countries 3 most important destination countries	(1) Malaysia (2) Taiwan (3) Hong Kong^1)^	(1) Malaysia (2) Saudi Arabia (3) Taiwan	(1) Malaysia (2) Saudi Arabia (3) Taiwan	(1) Malaysia (2) Taiwan (3) Hong Kong	(1) Hong Kong (2) Taiwan (3) Malaysia	(1) Hong Kong (2) Taiwan (3) Singapore

Sources: [17–19].

## Data Availability

The data analysed in this article are available in public domain and government offices website

## References

[1] Vignier N., Bouchaud O. (2018). Travel, migration and emerging infectious diseases. *The Journal of the International Federation of Clinical Chemistry and Laboratory Medicine*.

[2] Gushulak B. D., MacPherson D. W. (2004). Globalization of infectious diseases: The impact of migration. *Clinical Infectious Diseases*.

[3] Guadagno L. (2020). Migrants and the COVID-19 pandemic: An initial analysis. *Migration Research Series 2020*.

[4] World Bank (2020). COVID-19 crisis through a migration lens. *Migration And Development Brief 32*.

[5] World Health Organization (WHO) (2021). *Coronavirus Disease (COVID-19): How Is it Transmitted?” 2020*.

[6] World Health Organization (WHO) (2020). *Covid-19 Strategy Update*.

[7] World Health Organization (WHO) (2021). *Joint Statement from the International Coalition of Medicines Regulatory Authorities and World Health Organization*.

[8] (2020). The united nations office for the coordination of humanitarian affairs (OCHA) and the United Nations Resident Coordinator Office (RCO). https://indonesia.un.org/sites/default/files/2020-09/20200606-COVID19-MSRP-ENG.pdf.

[9] (2021). Indonesia COVID-19 Handling Taskforce. Indonesia’s COVID-19 data analysis. https://covid19.go.id/p/berita/analisis-data-covid-19-indonesia-update-26-desember-2021.

[10] Committee for Handling COVID-19 (2020). 3M and 3T one package for handling COVID-19. https://covid19.go.id/edukasi/masyarakat-umum/3m-dan-3t-satu-paket-penanganan-covid-19.

[11] Ministry of Health the Republic of Indonesia (2021). 5M during the COVID-19 pandemic in Indonesia. http://www.padk.kemkes.go.id/article/read/2021/02/01/46/5-m-dimasa-pandemi-covid-19-di-indonesia.html.

[12] Ministry of Health Republic Indonesia (2021). Public relations of the directorate general of disease control and control. “COVID-19 vaccination program begins, president the first person to receive COVID-19 vaccine injection”. http://p2p.kemkes.go.id/program-vaksinasi-covid-19-mulai-dilakukan-presiden-orang-pertama-penerima-suntikan-vaksin-covid-19/.

[13] International Labour Organization (ILO) (2021). *Labour and Social Trends in Indonesia 2014-2015: Strengthening Competitiveness and Productivity through Decent Work*.

[14] McAuliffe M., Kitimbo A., Abel G., Sawyer A., Klatt J. (2019). Migration and migrants: regional dimensions and developments. *World Migration Report 2020*.

[15] International Organization for Migration (IOM) (2021). *World Migration Report 2020*.

[16] World Bank (2017). *Indonesia’s Global Workers. Juggling Opportunities & Risks*.

[17] Indonesian National Labour Placement and Protection Agency (BNP2TKI) (2021). Indonesian migrant worker placement and protection data for the 2018 period. https://bp2mi.go.id/uploads/statistik/images/data_26-11-2019_data_12-03-2019_094615_Laporan_Pengolahan_Data_BNP2TKI_2018.pdf.

[18] Indonesian National Labour Placement and Protection Agency (BNP2TKI) (2021). Indonesian migrant worker placement and protection data for the 2019 period. https://bp2mi.go.id/uploads/statistik/images/data_19-02-2020_Laporan_Pengolahan_Data_BNP2TKI_2019.pdf.

[19] Indonesian Migrant Workers Protection Agency (BP2MI) (2022). Data on Indonesian migrant workers for the period 2021. https://bp2mi.go.id/uploads/statistik/images/data_11-04-2022_Laporan_Publikasi_Tahun_2021_Final_23022022.pdf.

[20] COVID-19 Handling Task Force (2022). Circular letter number 17, 2022 concerning foreign travel health protocols during the corona virus disease 2019 (COVID-19) pandemic. https://covid19.go.id/storage/app/media/Regulasi/2022/April/se-ka-satgas-nomor-17-tahun-2022-tentang-ketentuan-perjalanan-orang-dalam-negeri-pada-masa-pandemi-corona-virus-disease-2019-covid-19.pdf.

[21] Official Portal of Riau Islands Province (2021). 200 Indonesian migrant workers returned from Malaysia are infected with COVID-19. https://kepriprov.go.id/home/berita/5455.

[22] Ministry of Health of the Republic of Indonesia (2021). *Batam Class I Port Health Office. Handling COVID-19. Health Quarantine at the Entrance of the Country*.

[23] East Java Provincial Communication (2021). Total PMI infected with Covid-19 as many as 2,188 people. http://kominfo.jatimprov.go.id/read/pemulangan-pmi/total-pmi-terinfeksi-covid-19-sebanyak-2-188-orang.

[24] Aswatini A., Fitranita F., Rachmawati L., Noveria M. (2019). *Migration as an Investment for the Increased Competitiveness of Indonesian Migrant Workers in the Global Job market*.

[25] COVID-19.go.id (2022). COVID-19 distribution map. https://covid19.go.id/peta-sebaran-covid19.

[26] International Labour Organization (ILO) (2021). C097 - migration for employment convention (Revised), 1949 (No. 97). https://www.ilo.org/dyn/normlex/en/f?p=NORMLEXPUB:12100:0::NO::P12100_INSTRUMENT_ID:312242.

[27] United Nations (UN) (1990). International convention international convention on the protection of the rights of all migrant workers and members of their families.

[28] President of the Republic of Indonesia (2017). Number 18 of 2017 concerning the protection of Indonesian migrant workers. https://jdih.setkab.go.id/PUUdoc/175351/UU%20Nomor%2018%20Tahun%202017.pdf.

[29] Zimmerman C., Kiss L., Hossain M. (2011). Migration and health: a framework for 21st century policy making. *PLoS Medicine*.

[30] Greenaway C., Castelli F. (2019). Infectious diseases at different stages of migration: an expert review. *Journal of Travel Medicine*.

[31] Loganathan T., Rui D., Pocock N. S. (2020). Healthcare for migrant workers in destination countries: a comparative qualitative study of China and Malaysia. *BMJ Open*.

[32] The Government of the Republic of Indonesia (2020). *Government Regulation Number 10 of 2020 concerning Procedures for Placement of Indonesian Migrant Workers by the Indonesian Migrant Workers Protection Agency*.

[33] Riyadi R., Larasaty P. (2021). Factors that affect public compliance with health protocols in preventing the spread of COVID-19. *Prosiding Seminar Nasional Official Statistic 2020*.

[34] Wiranti A. S., Kusumastuti W. (2020). Determinants of Depok City community compliance with large-scale social restriction policies in preventing COVID-19. *Jurnal Kebijakan Kesehatan Indonesia*.

[35] Afrianti N., Rahmiati C. (2021). Factors affecting public compliance with the COVID-19 health protocol. *Jurnal Ilmiah STIKES Kendal*.

[36] Sari D. P., Atiqoh N. S. (2020). The relationship between public knowledge and compliance with the use of masks as an effort to prevent Covid-19 disease in Ngronggah. *Jurnal Ilmiah Rekam Medis dan Informatika Kesehatan*.

[37] Liem, Wang C., Dong C., Lam A. I. F., Latkin C. A., Hall B. J. (2021). Knowledge and awareness of COVID-19 among Indonesian migrant workers in the greater China region. *Public Health*.

[38] Indonesian Migrant Workers Protection Agency (2020). Indonesian migrant workers placement and protection data. https://bp2mi.go.id/uploads/statistik/images/data_03-03-2020_Laporan_Pengolahan_Data_BNP2TKI__JANUARI.pdf.

[39] Indonesian Migrant Workers Protection Agency (2020). Indonesian migrant workers placement and protection data. https://bp2mi.go.id/uploads/statistik/images/data_31-03-2021_LAPORAN_PENGOLAHAN_DATA_PMI_BULAN_FEBRUARI_TAHUN_2021_-_edit_19032021.pdf.

[40] Indonesian Migrant Workers Protection Agency (2020). Data and information centre (BP2MI). PMI placement and protection data for March 2020 period. https://bp2mi.go.id/uploads/statistik/images/data_22-04-2020_Laporan_Pengolahan_Data_BNP2TKI_MARET_(1)_(1).pdf.

[41] kawalcovid19.go.id (2021). Corona statistic. https://datastudio.google.com/u/0/reporting/fda876a7-3eb2-4080-92e8-679c93d6d1bd/page/h6oVB.

[42] Tapung M. M., Regus M., Payong M. R., Jelahut M. S. (2020). Socialization of health protocols during the COVID-19 pandemic and new normal for the people of Ruteng City (PKM with a critical phenomenological approach) 2020. http://ejournal.atmajaya.ac.id/files/journals/4/articles/1369/submission/1369-37-4107-1-2-20200722.docx.

[43] Aulia K. N. (2020). Increasing public awareness to pay attention to prokes (Health Protocols) in activities in the NeNo Era (New Normal) with PEPC media (Covid-19 prevention education posters) through wafagram media (WA, Facebook, and Instagram) in Kampung Padang Laban, Nagari Pasia Pelangai. https://osf.io/3upaj.

[44] International Labour Organization (ILO) (2020). *Ensuring Fair Recruitment During the Covid-19 Pandemic*.

[45] Thomson L. (2020). COVID-19: Guidance for labour recruiters to enhance migrant worker protection during the current health crisis. https://iris.iom.int/sites/default/files/COVID-19_Recruiter%20Guidance_Final_V1.pdf.

[46] Patunru A. A., Uddarojat R. (2015). Reducing the financial burden of Indonesian migrant workers. CIPS policy recommendations No. 1. https://repository.cips-indonesia.org/media/269-reducing-the-financial-burden-of-indones-bb2686ee.pdf.

[47] International Labour Organization (ILO) (2013). *10 Years Of Work On Labour Migration In Indonesia*.

[48] World Bank (2017). *Indonesia’s Global Workers: Juggling Opportunities and Risks. A World Bank Indonesia Report*.

[49] Susilo W. (2020). Education as an agenda for the protection of Indonesian migrant workers 2016. https://migrantcare.net/wp-content/uploads/2016/09/artikel_JP_migran_dan_pendidikan.pdf.

[50] SEMERU (2019). *Mampu Midline Study Thematic Report Theme 3: Access of Women Overseas Migrant Workers to Protective Services*.

[51] The Government of the Republic of Indonesia (2017). *Law Number 18 of 2017 concerning the Protection of Indonesian Migrant Workers*.

[52] Subhan H. (2012). Protection of Indonesian migrant workers in the pre-placement period, during placement, and after placement. https://www.bphn.go.id/data/documents/pkj_2012_-_5.pdf.

[53] International Finance Corporation (2020). Migrant workers Covid-19. EBRD-IFC briefing note. https://www.ebrd.com/documents/environment/ebrdifc-briefing-note.pdf.

[54] Machmudi M. I. (2020). 3 programs of the ministry of manpower related to mitigation of the Covid-19 pandemic. https://mediaindonesia.com/read/detail/326494-3-program-upaya-kemnaker-terkait-mitigasi-pandemi-covid-19.

[55] Ministry of Manpower of the Republic of Indonesia (2020). *Decree of the Minister of Manpower of the Republic of Indonesia Number 294 of 2020 Concerning the Implementation of the Placement of Indonesian Migrant Workers during the Adaptation Period of New Habits: 2020*.

[56] Indonesian Migrant Worker Placement and Protection Agency (BP2MI) (2020). List of CPMI examination health facilities. https://bp2mi.go.id/sarkes/indeks.

[57] Mery L., Rahmah A., Wulandari A. S. R. (2021). Regulation of the provision of covid-19 vaccination in Indonesia as the implementation of state obligationsin line with the Indonesian constitution. *SASI*.

[58] Indonesian Ministry of Health (2021). *The Degree of the General of Infection Prevention and Control MoH No 02.02/4/1/2021 on Technical Guideline of Vaccination for Management of the Corona Virus Diseases Pandemic 2019 (COVID-19) Indonesia*.

[59] ksp.go.id (2021). KSP will oversee vaccination for migrant workers. https://ksp.go.id/en/ksp-akan-kawal-vaksinasi-bagi-calon-pekerja-migran.html.

[60] Chia L. I. (2022). COVID-19: entry extended to more foreign labor. https://www.taipeitimes.com/News/front/archives/2022/02/08/2003772734.

[61] info.gov.hk (2021). Foreign domestic helpers who fully vaccinated in Indonesia and the Philippines may come to work in Hong Kong. https://www.info.gov.hk/gia/general/202108/26/P2021082600265.htm.

[62] Izan K. (2021). BP2MI facilitates PMI candidates to face COVID-19. https://www.antaranews.com/berita/2359734/bp2mi-fasilitasi-calon-pekerja-migran-jalani-vaksinasi-covid-19.

[63] jawapost.com (2021). Minister of manpower says the IMWs who were vaccinated by Sinovac were rejected by several countries. https://www.jawapos.com/ekonomi/25/08/2021/menaker-sebut-tki-yang-divaksin-sinovac-ditolak-beberapa-negara/.

[64] Khan A. H., Tirth V., Fawzy M. (2021). COVID‐19 transmission, vulnerability, persistence and nanotherapy: a review. *Environmental Chemistry Letters*.

[65] Wilson M. E. (2003). The traveller and emerging infections: sentinel, courier, transmitter. *Journal of Applied Microbiology Symposium Supplement*.

[66] Green A. D., Roberts K. I. (2000). Recent trends in infectious diseases for travellers. *Occupational Medicine*.

[67] Romdiati H., Noveria M., Bandiyono S. (2002). *Information Needs for Indonesian Migrant Workers: Case Studies in the Provinces of West Java, East Kalimantan, and Riau*.

[68] Castelli F., Sulis G. (2017). Migration and infectious disease. *Clinical Microbiology and Infections*.

[69] Taipei Economic and Cultural Center in India (2020). MOFA adjusts entry regulations for foreign nationals in response to worldwide efforts to resume economic activity and international exchanges following COVID-19 outbreak. https://www.roc-taiwan.org/in_en/post/4755.html.

[70] Ministry of the Interior National Immigration Agency (2021). CECC announces adjustments to regulations for foreign nationals entering Taiwan beginning January 1, 2021, in response to the continued spread of COVID-19 pandemic. https://www.immigration.gov.tw/5475/5478/141457/142068/248688/.

[71] Indonesia.go.id (2020). Protocol for the return of Indonesian citizens from abroad. https://indonesia.go.id/layanan/keimigrasian/ekonomi/protokol-kepulangan-wni-dari-luar-negeri.

[72] Benach J., Muntaner C., Delclos C., Menendez M., Ronquillo C. (2011). Migration and low-skilled workers in destination countries. *PLoS Medicine*.

[73] Marschke M., Vandergeest P., Havice E. (2020). COVID-19, instability and migrant fish workers in Asia. *Maritime Studies*.

[74] Hidayat H. (2017). Perlindungan hak tenaga kerja Indonesia di Taiwan dan Malaysia dalam perspektif hak asasi manusia. *Jurnal HAM*.

[75] Haley E., Caxaj S., George G., Hennebry J. L., Martell E., McLaughlin J. (2020). Migrant farmworkers face heightened vulnerabilities during COVID-19. *Journal of Agriculture, Food Systems, and Community Development*.

[76] Neef A. (2020). Legal and social protection for migrant farmworkers: lessons from COVID‐19. *Agriculture and Human Values*.

[77] Alahmad B., Kurdi H., Colonna K., Gasana J., Agnew J., Fox M. A. (2020). COVID-19 stressors on migrant workers in Kuwait: cumulative risk considerations. *BMJ Global Health*.

[78] Ngiam J. N., Chew N., Tham S. M. (2021). Demographic shift in COVID-19 patients in Singapore from an aged, at-risk population to young migrant workers with reduced risk of severe disease. *International Journal of Infectious Diseases*.

[79] Yi H., Ng S. T., Farwin A., Pei Ting Low A., Chang C. M., Lim J. (2021). Health equity considerations in COVID-19: geospatial network analysis of the COVID-19 outbreak in the migrant population in Singapore. *Journal of Travel Medicine*.

[80] Human Rights Working Group (HRWG) (2020). Impacts of COVID-19 on Indonesian migrant workers: From laid off from work, being unpaid, fear of arrested, to extra work without additional payment. https://hrwg.org/2020/05/10/siaran-pers-dampak-COVID-19-terhadap-pmi-dari-phk-gaji-tidak-dibayar-takut-ditangkap-sampai-kerja-ekstra-tanpa-tambahan-insentif/.

[81] Yazid S. (2022). Indonesia’s response to global recommendations on labour. Migration during a pandemic: muddling through priorities and needs. *Public Health in Asia during the COVID-19 Pandemic. Global Health Governance, Migrant Labour, and International Health Crises*.

[82] Indonesia.go.id (2019). Caring For Indonesian citizen portal abroad. https://indonesia.go.id/kategori/kependudukan/559/portal-peduliwni-di-luar-negeri.

[83] Davies A. A., Borland R. M., Blake C., West H. E. (2011). The dynamics of health and return migration. *PLoS Medicine*.

